# Target Deconvolution of Fenofibrate in Nonalcoholic Fatty Liver Disease Using Bioinformatics Analysis

**DOI:** 10.1155/2021/3654660

**Published:** 2021-12-26

**Authors:** Ali Mahmoudi, Alexandra E. Butler, Tannaz Jamialahmadi, Amirhossein Sahebkar

**Affiliations:** ^1^Department of Medical Biotechnology and Nanotechnology, Faculty of Medicine, Mashhad University of Medical Sciences, Iran; ^2^Royal College of Surgeons in Ireland Bahrain, Adliya, Bahrain; ^3^Department of Nutrition, Faculty of Medicine, Mashhad University of Medical Sciences, Mashhad, Iran; ^4^Biotechnology Research Center, Pharmaceutical Technology Institute, Mashhad University of Medical Sciences, Mashhad, Iran; ^5^Applied Biomedical Research Center, Mashhad University of Medical Sciences, Mashhad, Iran; ^6^School of Pharmacy, Mashhad University of Medical Sciences, Mashhad, Iran

## Abstract

**Background:**

Nonalcoholic fatty liver disease (NAFLD) is a prevalent form of liver damage, affecting ~25% of the global population. NAFLD comprises a spectrum of liver pathologies, from hepatic steatosis to nonalcoholic steatohepatitis (NASH), and may progress to liver fibrosis and cirrhosis. The presence of NAFLD correlates with metabolic disorders such as hyperlipidemia, obesity, blood hypertension, cardiovascular, and insulin resistance. Fenofibrate is an agonist drug for peroxisome proliferator-activated receptor alpha (PPAR*α*), used principally for treatment of hyperlipidemia. However, fenofibrate has recently been investigated in clinical trials for treatment of other metabolic disorders such as diabetes, cardiovascular disease, and NAFLD. The evidence to date indicates that fenofibrate could improve NAFLD. While PPAR*α* is considered to be the main target of fenofibrate, fenofibrate may exert its effect through impact on other genes and pathways thereby alleviating, and possibly reversing, NAFLD. In this study, using bioinformatics tools and gene-drug, gene-diseases databases, we sought to explore possible targets, interactions, and pathways involved in fenofibrate and NAFLD.

**Methods:**

We first determined significant protein interactions with fenofibrate in the STITCH database with high confidence (0.7). Next, we investigated the identified proteins on curated targets in two databases, including the DisGeNET and DISEASES databases, to determine their association with NAFLD. We finally constructed a Venn diagram for these two collections (curated genes-NAFLD and fenofibrate-STITCH) to uncover possible primary targets of fenofibrate. Then, Gene Ontology (GO) and KEGG were analyzed to detect the significantly involved targets in molecular function, biological process, cellular component, and biological pathways. A *P* value < 0.01 was considered the cut-off criterion. We also estimated the specificity of targets with NAFLD by investigating them in disease-gene associations (STRING) and EnrichR (DisGeNET). Finally, we verified our findings in the scientific literature.

**Results:**

We constructed two collections, one with 80 protein-drug interactions and the other with 95 genes associated with NAFLD. Using the Venn diagram, we identified 11 significant targets including LEP, SIRT1, ADIPOQ, PPARA, SREBF1, LDLR, GSTP1, VLDLR, SCARB1, MMP1, and APOC3 and then evaluated their biological pathways. Based on Gene Ontology, most of the targets are involved in lipid metabolism, and KEGG enrichment pathways showed the PPAR signaling pathway, AMPK signaling pathway, and NAFLD as the most significant pathways. The interrogation of those targets on authentic disease databases showed they were more specific to both steatosis and steatohepatitis liver injury than to any other diseases in these databases. Finally, we identified three significant genes, APOC3, PPARA, and SREBF1, that showed robust drug interaction with fenofibrate.

**Conclusion:**

Fenofibrate may exert its effect directly or indirectly, via modulation of several key targets and pathways, in the treatment of NAFLD.

## 1. Introduction

In recent decades, nonalcoholic fatty liver (NAFLD) has received greater attention from both healthcare professionals and the general public due to its increasing prevalence. NAFLD comprises a spectrum of liver disorders, from hepatic steatosis to nonalcoholic steatohepatitis (NASH) and, if unchecked, may progress to fibrosis and cirrhosis [1]. The hallmark of NAFLD is accumulation of fat deposits in hepatocytes, the presence of which correlates with metabolic disorders such as hyperlipidemia, obesity, hypertension, cardiovascular disease, and insulin resistance [2, 3]. The global prevalence of NAFLD is approximately ~25%, with the highest prevalence being found in the Middle East [4].

Despite the health burden it imposes, no definitive treatment for NAFLD has yet been determined, though various therapeutic approaches have been proposed. Lifestyle intervention and pharmacological interventions are the mainstays of treatment for patients with NAFLD.

As disruption of essential genes and proteins may lead to fatty liver diseases, identification of these targets enables drug discovery for treatment of NAFLD [5, 6]. Drug treatments include targeting caloric intake and disposal, inflammation, lipotoxicity, and cirrhosis [7–10]. One of the key drug targeting strategies is the modulation of hepatic fat accumulation, including targeting peroxisome proliferator-activator receptors and *de novo* lipogenesis [11]. Fenofibrate is an agonist drug for PPAR*α* and is principally used for treatment of hyperlipidemia in spite of the presence of statins and several newer lipid-lowering agents [12–15]. PPAR*α* is abundantly expressed in the liver and modulates various genes implicated in the catabolism of fatty acids [16]. However, it has recently been investigated in clinical trials for treatment of other metabolic disorders such as diabetes, cardiovascular disease, and NAFLD [17–19]. Additionally, reports suggest that fenofibrate could play a role in antioxidation, tumour apoptosis, anti-inflammation, and antifibrosis plus several other pliotropic effects [20–28]. Evidence from several clinical studies has shown that fenofibrate may provide benefit to patients with NASH/NAFLD [18, 29, 30].

While PPAR*α* is recognized to be the main target of fenofibrate, this drug may exert its effect via other genes and pathways that have not been well characterized to improve and possibly reverse NAFLD/NASH. Clinical investigation is already underway using fenofibrate for the treatment of NAFLD. Using bioinformatics tools and gene-drug, gene-diseases databases, we sought to explore other targets, interactions, and pathways involving fenofibrate and NAFLD. In Figure 1, we illustrate the overall strategy employed in this study.

## 2. Methods

### 2.1. Fenofibrate and Target Search

We first searched interactions of fenofibrate in the STITCH database (http://stitch.embl.de/) to explore essential protein targets. STITCH is a platform for diagnosis interaction between chemicals and proteins. Here, we considered the high confidence cut-off (0.700) and limited species only to Homo sapiens.

### 2.2. Exploring Important NAFLD Genes in DISEASES and DisGeNET Databases

Next, we investigated the protein targets identified in STITCH on curated targets in two databases, the DisGeNET database (https://www.disgenet.org/(and the DISEASES database (http://diseases.jensenlab.org/), to find their association with NAFLD. DisGeNET is a database that contains a collection of genes associated with specific diseases. That data is integrated from a variety of sources such as expert-curated repositories, the scientific literature and GWAS catalogs. DisGeNET currently covers more than 1,700 genes and 24,000 diseases and traits [31]. For association genes with NAFLD, 1,058 genes were registered in this database. Curated data contain seven primary resources: UNIPROT, ORPHANET, CTD, GENOMICS ENGLAND, CLINGEN, PSYGENET, and CGI. To achieve a curated dataset from DisGeNET, we used a plugin in the cystoscope to construct curated sources targets for NAFLD. DISEASES database is a weekly updated database that comprises diseases and gene relations from different resources, including manually curated literature, text mining, cancer mutation data, and genome-wide association research [32]. We extracted the targets from the available resources, including experiments and manually curated literature associated with NAFLD.

### 2.3. Venn Diagram to Obtain Important Fenofibrate Interaction Protein Targets in NAFLD

We finally created a Venn diagram (http://bioinformatics.psb.ugent.be/webtools/Venn/) for these two collections (curated genes-NAFLD and fenofibrate-STITCH) to find important targets of fenofibrate beyond the conventionally recognized targets.

### 2.4. Gene Ontology Pathway Enrichment Analyses for Target Proteins of Fenofibrate

Gene ontology (GO) enrichment is a popular procedure used to interpret genes and stratify them in three major categories, those that contribute to molecular function (MF), biological process, (BP) or cellular component (CC). GO was analyzed for important targets obtained from the Venn diagram using the Gene Ontology resource with the web address: http://geneontology.org. Additionally, KEGG was analyzed using the Enrichr database with the web address: https://maayanlab.cloud/Enrichr/. The KEGG pathway is a comprehensive database that maps pathways according to their metabolic interrelationships. In GO and KEGG analyses, the *P* value < 0.01 was considered the cut-off criterion. We also analyzed the enrichment pathways using the wikipathways plugin in Cytoscape version 3.8.2. A *P* value < 0.01 was considered the cut-off criterion. In addition, we estimated the specificity of obtained targets with NAFLD and investigated them in disease-gene associations (STRING) and EnrichR (DisGeNET).

## 3. Results

### 3.1. Protein Target Interaction with Fenofibrate in the STITCH Database

Screening fenofibrate in the STITCH database with high confidence (0.7) identified 80 protein targets. The drug-protein interaction was visualized on Cytoscape (Figure 2(a)).

### 3.2. Discovering Curated NAFLD Genes

The curated data DisGeNet plugin on Cytoscape and DISEASES database identified 95 genes associated with NAFLD. All the data are visualized with Cytoscape software (Figure 2(a)).

### 3.3. Overlap of Fenofibrate Targets on the STITCH and Curated NAFLD Genes Visualized Using a Venn Diagram

A Venn diagram of the two created datasets revealed eleven candidates, including SREBF1, SCARB1, LDLR, PPARA, VLDLR, LEP, MMP1, GSTP1, SIRT1, APOC3, and ADIPOQ (Figure 2(b)) that may be directly or indirectly affected by fenofibrate. The scoring based on DisGeNET is shown in Table 1. Based on the database algorithm (genes-disease associate score), five targets (LEP, SIRT1, ADIPOQ, PPARA, and SREBF1) are the most important in NAFLD.

### 3.4. GO and KEGG Enrichment Analyses of Protein Targets of Fenofibrate

GO analysis of the 11 identified protein targets demonstrated major involvement in the regulation of the lipid biosynthetic process, the lipid metabolic process, and the lipid metabolic process under biological process (Table 2). This analysis additionally showed that these protein targets were chiefly involved in lipoprotein particle receptor activity, protein-lipid complex binding, and lipoprotein particle binding under the molecular function category. Furthermore, cellular components included the lipoprotein particle, plasma lipoprotein particle, and protein-lipid complex (Table 2).

In KEGG enrichment, we observed several biological pathways. The highest *P* value pathways included the PPAR signaling pathway and the AMPK signaling pathway (Table 3).

The DISEASES database, based on the STRING algorithm, and the DisGeNETdatabase, based on the EnrichR algorithm, revealed the association of 11 of the identified proteins with NAFLD and its advanced form NASH, these diseases ranking in the top three in both databases (Table 4). Therefore, their close relationship with fatty liver disease was confirmed.

In contrast, by setting the cut-off for the STITCH database to 0.9, we identified 22 protein interactions with fenofibrate. PPARA, with a score of 0.995, was the highest ranked protein target in this PPI network. SERPINE1, CCL2, CRP, and VCAM1, with a score of 0.984, were the next most significant protein targets after PPARA in the PPI network. Moreover, protein targets were restricted to three significant genes in the Venn diagram with a preprepared curated disease database. Those three protein targets were SREBF1, APOC3, and PPARA.

We also visualized the degree of connection with high confidence (0.7) of the protein targets to fenofibrate in the NAFLD pathway. The more intense color indicates greater interaction (based on the STITCH score) (Figure 3). The pathways are constructed based upon the wikipathway dataset with access number WP4396 using the Cytoscape plugin.

## 4. Discussion

NAFLD is a highly prevalent chronic liver disease, comprising a spectrum of liver pathologies, from hepatic steatosis to nonalcoholic steatohepatitis (NASH), and may progress to liver fibrosis and cirrhosis. [33]. NAFLD is commonly identified as a multifactorial disease with interaction amongst risk factors and susceptibility genes that play a central role in the development and phenotype of NAFLD [34]. Consequently, identifying those targets and employing suitable therapeutic agents are important steps in improving treatment modalities. Fenofibrate is a drug that is proven for treatment of hyperlipidemia. Additionally, some studies have shown positive results with fenofibrate for the treatment of NAFLD. Fenofibrate has been shown to improve NAFLD in various research studies using cell lines and animal models, as well as in clinical studies in humans. For example, it has been reported that fenofibrate reduces fat content in the liver, reverses hepatic steatosis and fibrosis, and alleviates pathological liver changes in animals with NAFLD [35, 36]. A clinical study revealed that liver enzymes, blood pressure, and body mass index considerably improved, and that treatment with fenofibrate was advantageous due to its beneficial effects in patients with NAFLD [37]. Moreover, an *in vitro* study on steatotic HepaRG cell lines demonstrated the effect of fenofibrate on ameliorating hepatic steatosis [38]. The mechanism that has been widely purported is through fenofibrate's antagonistic effect on PPAR*α*. However, in our study, according to the results of prediction and its interactions directly and indirectly with other targets using bioinformatics software, the mechanism of fenofibrate's mode of action may be broader than an exclusive role of PPAR*α* antagonism. Here, we investigated and analyzed those predictions in other disease-genes, drug-protein databases and biological pathways to understand in greater depth the possible effects of fenofibrate in NAFLD.

In the work presented here, we first searched significant prediction protein interaction with high confidence for fenofibrate. Then, we probed protein interaction in association with fatty liver disease and selected the most relevant targets. In so doing, we identified 11 significant targets, including LEP, SIRT1, ADIPOQ, PPARA, SREBF1, LDLR, GSTP1, VLDLR, SCARB1, MMP1, and APOC3, and we then evaluated their biological pathways. Based on gene ontology, most of the targets were involved in lipid metabolism, and KEGG enrichment pathways showed PPAR signaling pathway, AMPK signaling pathway, and NAFLD as the most significant pathways. The targets we found among the authentic disease databases were more specific to fatty liver disease (steatosis and steatohepatitis) than other diseases in these databases. We finally identified three important significant genes, APOC3, PPARA, and SREBF1, showing robust drug interaction with fenofibrate.

The PPAR signaling pathway is comprised of three receptor subtypes, alpha, gamma, and beta/delta, which are activated by fatty acids and their derivatives. Each subtype is encoded by a separate gene. PPAR-alpha is important for lipid metabolism in the liver and functions in the clearance of circulating and cellular lipids. The function of PPAR-gamma is in the induction of adipocyte differentiation which causes increased uptake of blood glucose. PPAR-beta/delta also contributes to lipid oxidation and cell proliferation [39, 40]. By applying different agonists to this pathway, research has shown a decrease in triglycerides, modulation of circulating glucose, and an elevation in HDL [41–43]. In this way, these agonists could ameliorate NAFLD. The PPAR signaling pathway contains various genes that show enrichment in our study: based on KEGG analysis, enrichment of MMP1, ADIPOQ, APOC3, and PPARA revealed that this pathway shows a robust interaction with fenofibrate (*P* value: 5.586*e* − 8). PPAR-alpha is principally present in the liver, while PPAR-gamma is mainly expressed in adipose tissue [44]. Expression of PPAR-gamma has been reported to be significantly increased in the liver of patients and animal models with NAFLD [45–47]. This elevation might be a consequence of the expression of the adipogenic genes that induce lipid accumulation in the liver of these patients and animals with NAFLD [48].

AMPK (adenosine monophosphate-activated protein kinase) has serine/threonine kinase as its catalytic alpha subunit and beta/gamma as its regulatory subunit [49]. This pathway is involved in lipid metabolism and energy sensing, regulating glucose in numerous tissue such as the liver [50]. In our study, enrichment of SREBF1, LEP, ADIPOQ, and SIRT1 genes was found, and the AMPK pathway was significantly (*P* value: 3.937*e* − 7) shown to be influenced by fenofibrate. AMPK is regulated by phosphorylation and dephosphorylation via kinases. Activation of AMPK results in an orderly adjustment of energy balance in metabolic processes. It increases fatty acid oxidation and reduces triglyceride and cholesterol production, consequently decreasing fat accumulation [51]. Due to these actions, this pathway is considered to be a therapeutic target for a metabolic disorder such as NAFLD [52, 53]. Activation of AMPK is connected to improvement in liver inflammation and metabolism in NAFLD [54, 55]. Additionally, several studies have demonstrated that AMPK signaling pathways are involved in liver steatosis and steatohepatitis [56]. Research in 2014 indicated that fenofibrate could modulate AMPK signaling and thereby exert its therapeutic effect [57].

Research has demonstrated that lipid accumulation in the liver involves a reduction in fatty acid oxidation and VLDL secretion and upregulation of adipogenic and lipogenic pathways, through which lipoprotein particles deliver fatty acids to the liver [58]. Based on the gene ontology analysis (Table 2), important genes in these pathways operate at the three stages of biological, molecular, and cellular components and could be influenced,with high confidence, by fenofibrate.

PPARA is one of the most important genes in NAFLD and that it interacts with fenofibrate is well established. As shown in our analysis, PPARA had the highest score for interaction with fenofibrate. Moreover, its role in NAFLD was also investigated, again showing a high score. However, our aim was to investigate targets other than PPARA and, hence, here, we discuss the possible influence of other targets with fenofibrate and their role in the pathogenesis of NAFLD.

SREBF1 is an essential factor in modulation of lipogenesis [59]. In models of NAFLD, SREBF1 was downregulated following induction of steatosis [60]. However, in patients with NAFLD, SREBF1 was reported to be significantly higher than the control group [61]. Moreover, enhancing cleavage of SREBF2 was shown to boost lipogenesis [62]. A recent study revealed that SREBF1 is activated through zinc finger and BTB domain-containing 7A (ZBTB7A), which causes lipid accumulation and progression of NAFLD [63]. Numerous studies have reported that SREBF1 is a potential target influencing NAFLD, as evidenced by administration of various interval treatments [64–66]. A recent study in 2021 by Elsayed et al. indicated that SREBF1 elevation is a risk factor in the progression of NAFLD and that, following treatment of NAFLD, this gene was downregulated. Fenofibrate, by direct binding of PPARA to the DR1 motif of SREBF1, may induce SREBF1 expression [67]. A TRANSFAC analysis revealed that after treatment with fenofibrate, MuRF1 -/- genes commonly had a SREBF1 promoter region [68]. Other researchers showed that fenofibrate could promote CREBH products and reduce SREBF1 levels [69]. Of note, in our study (Table 1), SREBF1 had the second highest score for interaction with fenofibrate after PPARA and showed a strong relationship to NAFLD.

ADIPOQ (adiponectin) is an adipose-derived plasma protein that functions in hepatic lipoprotein-lipid metabolism [70]. Several pieces of evidence indicate that diverse polymorphisms in ADIPOQ may increase susceptibility to NAFLD [70, 71]. One study reported that the ADIPOQ methylation rate in rats with NAFLD was higher than in control animals [72]. ADIPOQ in NAFLD patients is a risk factor for progression to liver cancer, and ADIPOQ is significantly decreased in patients with liver metastases [73]. Research has shown that the methylation rate of ADIPOQ in the NAFLD rat model is higher than in controls; further, alteration of the methylation rate pattern of ADIPOQ was hepatoprotective in the NAFLD group [72]. Another study reported that the level of ADIPOQ in serum is lower in NAFLD than controls and was associated with increased liver enzymes and lipid profile changes in patients with NAFLD [74]. Several studies have suggested that fenofibrate may modulate the level of adiponectin in diabetes, cardiomyocyte hypertrophy, and hypertriglyceridemia [75–77]. Fenofibrate caused an increase in serum adiponectin [78]. Fenofibrate may enhance adiponectin expression through modulation of PPAR-alpha expression [76]. Fenofibrate may also promote adiponectin through the AMPK signaling pathway [79]. Other researchers claimed that fenofibrate significantly reduced proinflammatory biomarkers and ameliorated adipocytokines through induction of adiponectin [80]. In our study, ADIPOQ was one of the highest scoring targets in terms of drug interactions with fenofibrate and an association with NAFLD.

LEP (leptin) is a polypeptide hormone that interacts with its receptor lepRb [81]. In a number of studies, the pathogenesis of leptin in NAFLD has been investigated. The level of leptin significantly increased in the serum of patients with NAFLD and in animal models of the disease and possibly normalized with the development of hepatocyte steatosis [81–84]. Leptin may be implicated in steatosis progression via activation of the PI3-K/Akt kinase pathway via OB-R [85, 86]. Numerous studies have reported that fenofibrate affects LEP expression. Previous clinical studies have also shown that fenofibrate affects the level of leptin in patients with dyslipidemia and hypertriglyceridemia and improves insulin sensitivity [80, 87–89]. Furthermore, LEP scored highly in both the drug interaction and diseases-relation interrogation, scoring 0.829 and 0.4, respectively.

SIRT1 is one of the important genes identified in the pathogenesis of fatty liver disease. SIRT1, a NADPH-dependent deacetylase, has a vital function in cellular processes, including stress response, transcriptional regulation, longevity, and apoptosis [90]. A number of reports implicate miRNAs that target SIRT1 in the pathogenesis of NAFLD [91–93]. SIRT1 is significantly downregulated in NAFLD [94], and interventions aimed at modulating SIRT1 have shown positive effects on NAFLD [95–99]. Fenofibrate can indirectly upregulate SIRT1 and repress hepatocyte apoptosis via SIRT1 and FoxO1 [100, 101]. The upregulation of SIRT1 may be accomplished through AMPK in TNF-*α*-stimulated adipocytes [102]. Another study showed that fenofibrate promotes SIRT1 expression, causing a reduction in NF-*κ*B activity [103]. Fenofibrate has been shown to affect a reduction in fat deposition and to alleviate inflammation through SIRT1-dependent pathways [104, 105]. In our study, SIRT1 was identified as one of critical gene associations with NAFLD and exhibited a robust interaction with fenofibrate.

Apolipoprotein C3 (APOC3) is a small protein on the surface of lipoprotein particles and has a vital role in regulating triglyceride metabolism. APOC3 has a potent inhibitor effect on lipoprotein lipase [106]. A study by Pavia et al. indicated that overexpression of APOC3 results in pathological features in the liver similar to NAFLD such as inflammation, hepatocyte apoptosis, oxidative stress, and increased liver lipid content [107]. It has been reported that fenofibrate significantly reduces the level of APOC3. In this study, fenofibrate demonstrated a robust interaction with APOC3 based upon the STITCH score (high confidence: 0.944). APOC3 placed eleventh in the curated diseases database (Table 1), indicating it may have a role in the pathogenesis of NAFLD.

MMP (matrix metalloproteinase) is a proteinase that can degrade components of the extracellular matrix and diverse nonmatrix proteins. MMPs have been shown to be involved in the pathogenesis of liver diseases [108]. MMP1 may have a role in the progression of NAFLD to NASH and then to liver fibrosis [109, 110]. Two studies demonstrated that fenofibrate could decrease MMP1 and that it repressed the enzymic actions of MMP2 and MMP9 [57, 111]. MMP1, as demonstrated here, shows significant interaction with fenofibrate (high confidence score based on STITCH of 0.872).

SCARB1 (scavenger receptor class B, type I) is a high-density lipoprotein (HDL) receptor that facilitates uptake of cholesterol (Cho) from HDL to hepatocytes [112, 113]. Recently, it has been suggested that SCARB1 may be associated with NAFLD [114] and several studies suggest that fenofibrate affects SCARB1 [115–117]. Those studies have proposed that fenofibrate may enhance the degradation of SCARB1 in a postendoplasmic reticulum or postplasma membrane compartment [115]. However, it is possible that fenofibrate does not directly inhibit SCARB1 [118]. The posttranscriptional regulation of fenofibrate may be dependent upon PPAR*α* expression [117]. According to our data shown in Table 1, SCARB1 is one of the top predicted targets for fenofibrate interaction, and investigation in the curated database revealed its relationship to NAFLD.

LDLR (low-density apolipoprotein receptor) is a mediator for cholesterol uptake in cells. It plays a crucial function in the clearance of cholesterol by the liver [119]. LDLR deficient rodents have been used to establish models of NAFLD [120, 121]. In those models, elevations in hepatic neutral and hepatic proinflammatory oxylipins were observed [122]. Some patients with NAFLD have been found to have mutations in LDLR genes [123]. Numerous studies have also demonstrated that fenofibrate affects LDLR expression; fenofibrate elevated hepatic LDLR via Akt phosphorylation and maturation of SREBP2 [124]. As shown in Table 1, LDLR was one of the eleven important genes that interacted with fenofibrate and was associated with NAFLD.

VLDLR (very-low-density lipoprotein receptor) has a critical role in modulating serum triglycerides and NAFLD progression [125]. Research on a mouse NAFLD model has demonstrated that antagonism of PPAR*β*/*δ* may regulate VLDLR and influence the serum triglyceride level and progression of NAFLD [125]. Studies have indicated that fenofibrate could influence VLDLR, but its mechanism and exact effect are still unclear [126, 127].

GSTP1 (glutathione S transferase Pi 1) is a gene that has a vital role in antioxidant defense through detoxifying foreign substances and inactivating byproducts of oxidative stress [128, 129]. Moreover, several studies published that some polymorphisms of GSTP1 are frequent in patients with NAFLD [130, 131]. The effect of fenofibrate on GSTP1 has not been studied in depth, and the available results are contradictory [132–136]. However, GSTP1 was one of eleven significant targets identified in our study and listed in Table 1.

## 5. Conclusion

In this study, we investigated the effect of fenofibrate on important targets in NAFLD. Our results indicate that fenofibrate may influence essential genes in NAFLD via an, as yet, undetermined mechanism. Fenofibrate could therefore benefit patients by preventing progression or even reversing severity of NAFLD. According to the results presented here, fenofibrate significantly influences essential biological pathways, including lipid metabolic processes via the PPAR signaling pathway and the AMPK signaling pathway. Notably, those targets have been validated as featuring in the pathogenesis of NAFLD. Consequently, fenofibrate may offer a significant benefit to patients with NAFLD, though further molecular and clinical investigation is required.

## Figures and Tables

**Figure 1:** A comprehensive diagram illustrating the investigative strategy undertaken in the present study.

**Figure 2:** (a) Curated disease-gene database and fenofibrate-protein interaction visualized with Cytoscape software. (b) Venn diagram of the two datasets comprising curated disease-gene database and fenofibrate-protein interaction.

**Figure 3:** Visualizing protein interactions with fenofibrate in the NAFLD pathway with high confidence (0.7) based on the STITCH score. The intensity of color illustrates the degree of interaction of fenofibrate with the targets.

**Table 1:** The relationship of genes associated with NAFLD that are targets of fenofibrate (http://www.disgenet.org/).

Gene	UniProt	Gene full name	Protein class	DSI g	Score gda	STITCH score
*LEP*	P41159	Leptin	Plasma protein	0.349	0.4	0.829
*SIRT1*	Q96EB6	Sirtuin 1	Epigenetic regulator	0.378	0.4	0.8
*ADIPOQ*	Q15848	Adiponectin, C1Q, and collagen domain containing	Transporter	0.376	0.4	0.884
*PPARA*	Q07869	Peroxisome proliferator-activated receptor alpha	Nuclear receptor	0.432	0.4	0.995
*SREBF1*	P36956	Sterol regulatory element binding transcription factor 1	Plasma protein, transcription factor	0.518	0.38	0.962
*LDLR*	P01130	Low-density lipoprotein receptor	Plasma protein	0.449	0.37	0.816
*GSTP1*	P09211	Glutathione S-transferase pi 1	Enzyme	0.383	0.33	0.8
*VLDLR*	P98155	Very-low-density lipoprotein receptor	Plasma protein	0.558	0.31	0.823
*SCARB1*	Q8WTV0	Scavenger receptor class B member 1	Receptor	0.559	0.3	0.853
*MMP1*	P03956	Matrix metallopeptidase 1	Enzyme	0.385	0.3	0.872
*APOC3*	P02656	Apolipoprotein C3	Plasma protein	0.531	0.1	0.944

Score gda (genes-disease associate score): the gda score is based on supporting evidence that has been collated from different sources as regards the association of genes and diseases. The gda score ranges from 0 to 1, so the closer this range is to 1 indicates a stronger the association between gene and disease. DSI (disease specificity index): a gene may be associated with numerous diseases. This index indicates the specificity of diseases to a particular gene. The index ranges from 0 to 1. A gene with many disease associations has a zero DSI index and, by contrast, a gene associated with just one disease has a DSI of 1. STITCH score: the STITCH score is a confidence indicator of how likely it is that STITCH will correctly evaluate an interaction based on evidence from preceding studies and predictions. Scores range from 0 to 1, with one being the highest confidence level for interaction and 0 being the highest level of uncertainty. A score of 0.5, for example, indicates that the interaction could be 50% false (i.e., a false positive).

**Table:** (a) Biological process (GO)

Accession	Pathway description	Gene count	*P* value	FDR
GO:0046890	Regulation of lipid biosynthetic process	7	7.07*E*^−13^	1.11*E*^−08^
GO:0019216	Regulation of lipid metabolic process	8	7.10*E*^−13^	5.59*E*^−09^
GO:0034381	Llasma lipoprotein particle clearance	5	1.76*E*^−12^	9.25*E*^−09^
GO:0006629	Lipid metabolic process	10	3.39*E*^−12^	1.33*E*^−08^
GO:1905952	Regulation of lipid storage	5	6.75*E*^−11^	2.13*E*^−07^

**Table:** (b) Molecular function (GO)

	Pathway description	Gene count	*P* value	FDR
GO:0030228	Lipoprotein particle receptor activity	3	1.50*E*^−07^	7.32*E*^−04^
GO:0044877	Protein-lipid complex binding	3	5.57*E*^−07^	1.36*E*^−03^
GO:0071813	Lipoprotein particle binding	3	5.57*E*^−07^	9.07*E*^−04^
GO:0030229	Very-low-density lipoprotein particle receptor activity	2	3.88*E*^−06^	4.75*E*^−03^
GO:0005041	Cargo receptor activity	3	1.50*E*^−07^	7.32*E*^−04^

**Table:** (c) Cellular component (GO)

	Pathway description	Gene count	*P* value	FDR
GO:1990777	Lipoprotein particle	3	1.11*E*^−06^	2.20*E*^−03^
GO:0034358	Plasma lipoprotein particle	3	1.11*E*^−06^	1.10*E*^−03^
GO:0032994	Protein-lipid complex	3	1.38*E*^−06^	9.16*E*^−04^
GO:0034361	Very-low-density lipoprotein particle	2	5.95*E*^−05^	2.96*E*^−02^
GO:0034385	Triglyceride-rich plasma lipoprotein particle	2	6.51*E*^−05^	2.59*E*^−02^

FDR (false discovery rate): FDR is a stringent statistical method allowing multiple comparisons while preserving a low false-positivity rate.

**Table 3:** KEGG pathways for 11 critical genes interact with fenofibrate.

Num.	KEGG			
	Pathway name	Genes	Gene count	*P* value
1	PPAR signaling pathway	MMP1, ADIPOQ, APOC3, PPARA	4	5.586*e* − 8
2	AMPK signaling pathway	SREBF1, LEP, ADIPOQ, SIRT1	4	3.937*e* − 7
3	Nonalcoholic fatty liver disease	SREBF1, LEP, ADIPOQ, PPARA	4	0.000001098
4	Cholesterol metabolism	SCARB1, APOC3, LDLR	3	0.000002392
5	Adipocytokine signaling pathway	LEP, ADIPOQ, PPARA	3	0.000006357

**Table:** (a) Disease-gene associations (STRING)

Identifier	Primary name	FDR
DOID:0080208	Nonalcoholic fatty liver disease	4.23*e* − 07
DOID:11716	Prediabetes syndrome	0.0037
DOID:0080547	Nonalcoholic steatohepatitis	0.0058

**Table:** (b) DisGeNET (EnrichR)

	Primary name	*P* value
1	Nonalcoholic fatty liver disease	1.598*e* − 17
2	Nonalcoholic steatohepatitis	6.748*e* − 17
3	Acute coronary syndrome	4.157*e* − 16

## Data Availability

Data associated with this study are available from the authors upon a reasonable request.
